# CREB1 Transcriptionally Activates LTBR to Promote the NF-*κ*B Pathway and Apoptosis in Lung Epithelial Cells

**DOI:** 10.1155/2022/9588740

**Published:** 2022-09-09

**Authors:** Zhengyun Hu, Guoping Zhou

**Affiliations:** ^1^Department of Pediatrics, The First Affiliated Hospital of Nanjing Medical University, Nanjing 210029, China; ^2^Department of Pediatrics, Shanghai Songjiang District Central Hospital, Shanghai 201600, China

## Abstract

Bronchopulmonary dysplasia (BPD) is a prevalent chronic pediatric lung disease. Aberrant proliferation and apoptosis of lung epithelial cells are important in the pathogenesis of BPD. Lymphotoxin beta receptor (LTBR) is expressed in lung epithelial cells. Blocking LTBR induces regeneration of lung tissue and reverts airway fibrosis in young and aged mice. This study is aimed at revealing the role of LTBR in BPD. A mouse model of BPD and two *in vitro* models of BPD using A549 cells and type II alveolar epithelial (ATII) cells were established by exposure to hyperoxia. We found that LTBR and CREB1 exhibited a significant upregulation in lungs of mouse model of BPD. LTBR and CREB1 expression were also increased by hyperoxia in A549 and ATII cells. According to results of cell counting kit-8 assay and flow cytometry analysis, silencing of LTBR rescued the suppressive effect of hyperoxia on cell viability and its promotive effect on cell apoptosis of A549 and ATII cells. Bioinformatics revealed CREB1 as a transcriptional factor for LTBR, and the luciferase reporter assay and ChIP assay subsequently confirmed it. The NF-*κ*B pathway was regulated by LTBR. CREB1 induced LTBR expression at the transcriptional level to regulate NF-*κ*B pathway and further modulate A549 and ATII cells viability and apoptosis. In conclusion, this study revealed the CREB1/LTBR/NF-*κ*B pathway in BPD and supported the beneficial role of LTBR silence in BPD by promoting viability and decreasing apoptosis of lung epithelial cells.

## 1. Introduction

Bronchopulmonary dysplasia (BPD), initially described by Northway et al., is caused by oxygen supply and mechanical ventilation in premature infants with severe respiratory distress syndrome [1]. According to the latest article by Higgins et al. [2], a premature infant with BPD has persistent parenchymal lung disease, confirmed by radiography, and at 36 weeks postmenstrual age requires 1 of the following: FiO_2_ ranges/oxygen levels/O_2_ concentrations for more than three consecutive days to maintain arterial oxygen saturation ranging between 90% and 95%. A review research concludes that BPD may be caused by various factors like premature birth, fetal growth restriction, mechanical ventilation, oxygen toxicity, inflammation, and genetic susceptibility [3]. Despite prenatal usage of glucocorticoid [4], pulmonary surfactant [5], and moderate ventilation strategy [6] were developed to decrease the incidence rate or prolong the survival rate of BPD in premature infants, there is no single effective prevention measures or treatments for BPD [7]. Thus, it is particularly important to explore the potential molecular mechanism of BPD.

BPD is a chronic disease featured by disrupting the alveolar together with microvascular development of the peripheral lung. The regeneration or induced growth of type II alveolar epithelial (ATII) cells has been the focus feature of lung regeneration research [8]. Thus, exploring the potential mechanism underlying ATII cells is vital for BPD development and treatment.

Activation of the LT*β* receptor (LTBR) signaling in ATII cells induces kinase NIK through nonclassical nuclear factor-kappaB (NF-*κ*B) signaling. Blocking LTBR signaling limits broncho-associated lymphoid tissue formation and reduces alveolar epithelial cell apoptosis, thereby driving alveolar regeneration [9]. LTBR signaling pathway plays an essential role in lymphatic organogenesis, tissue regeneration, organ development, tumorigenesis, and immune response to pathogen infection [10]. LTBR mRNA shows high levels in ATII cells in lungs of mice exposed to chronic cigarette smoke [9]. LTBR expression can be detected by immunofluorescence staining in A549 [11], a continuous tumor cell line with properties of ATII cells from lung cancer tissues.

Transcription factors respond to stimuli of the external environment or signals at different stages of development, activate or inhibit gene transcription, and thus control the expression of different genes. It is very important to identify key transcription factors in BPD. cAMP responsive element binding protein 1 (CREB1) regulates late-stage lung development in mammals [12]. CREB1 is activated in the lungs in response to alveolar hypoxia and is crucial for maintaining low pulmonary vascular resistance and normal alveolar structure under hypoxia [13]. It has been revealed that long noncoding RNA (lncRNA) MALAT1 regulates STING transcription in neonates with BPD through transcription factor CREB1 [14].

The NF-*κ*B signaling plays a crucial role in cell survival, differentiation, and innate immunity [15]. NF-*κ*B dimers are not active in the cytoplasm of cells related to a suppressive protein, I*κ*B. Under the conditions of cytokines, growth factors, or bacterial products, I*κ*B kinases IKK-*α* and -*β* activate NF-*κ*B, leading to I*κ*B phosphorylation and degradation. Clearance of I*κ*B allows translocation of NF-*κ*B complexes into the nucleus and modulates a variety of downstream targets that affect inflammation, cell adhesion, and cell survival [16]. Many studies have pointed NF-*κ*B-mediated gene modulation is implicated in the pathogenesis of BPD [17].

This study is aimed at evaluating the expression of LTBR in the BPD lung injury mouse model *in vivo* and its role in the apoptosis of lung epithelial cells *in vitro*. Hyperoxia-stimulated A549 and ATII cells were used as the *in vitro* model of BPD [18, 19]. The potential binding of CREB1 on LTBR promoter as well as the downstream NF-*κ*B pathway was assessed, providing new ideas for understanding the pathogenesis of BPD.

## 2. Materials and Methods

### 2.1. Hyperoxia Murine Models

Neonatal C57BL/6 mice of both sexes (Shanghai SLAC Laboratory Animal Co., Ltd., Shanghai, China) were used for establishing the model of BPD. Animal studies were conducted in compliance with the ARRIVE guidelines under the approval of the animal care and ethic committee of First Affiliated Hospital of Nanjing Medical University. Mice were housed under controlled standard conditions (21–23°C, 50–60% humidity, 12 h light/12 h dark cycle). Neonatal mice in the normoxia group were exposed to room air and fed by lactating mice. Mice were randomly divided into the BPD model group (*n* = 8) or the control group (*n* = 8). To establish the BPD model, mice were exposed to 100% O_2_ in a medium-sized airtight polypropylene chamber on postnatal days 1-4, followed by recovering for 10 days [19]. Neonatal pups were given adequate nutrition by lactating dam during experimental time to avoid death. At postnatal day 14, mice were euthanatized by intraperitoneal injection of 1 ml of 2.5% avertin [20], and lung tissues were dissected for the following assays.

### 2.2. Real-Time PCR

Total RNA was extracted from mice lungs or cultured A549 and ATII cells using the TRIzol regent (Invitrogen, USA) and dissolved in RNase-free water. Reverse transcription of total RNA into cDNA was performed using a High-Capacity cDNA Reverse Transcription Kit (#4368813; Applied Biosystems, USA). Next, the QuantiFast SYBR® Green PCR Kit (QIAGEN) was used for a rapid and specific quantitative detection of target cDNA. PCR analysis was performed on a LightCycer®480II Instrument, 96-well block (#05 015 278 001; Roche, USA). LTBR or CREB1 expression was calculated using the 2^-*ΔΔ*ct^ method [21] and was normalized to GAPDH expression. All qPCR primers in this study were listed as follows:

Mouse LTBR, forward, 5′-TGAACACTGGAACCATCTC-3′; reverse, 5′-ACACTCATTGTCCAGATACAC-3′.

Human LTBR, forward, 5′-GAAGGGTAACAACCACTGC-3′; reverse, 5′-CTTGGTTCTCACACCTGGT-3′.

Mouse CREB1, forward, 5′-GAAGAGGAGACTTCAGCCC-3′; reverse, 5′-TAATGGCAATGTACTGCCCA-3′.

Human CREB1, forward, 5′-ATGCAGCTGTAACAGAAGC-3′; reverse, 5′-CATAGATACCTGGGCTAATGTG-3′.

Mouse GAPDH, forward, 5′-ACTCTTCCACCTTCGATGC-3′; reverse, 5′-CCGTATTCATTGTCATACCAGG-3′.

Human GAPDH, forward, 5′-TCAAGATCATCAGCAATGCC-3′; reverse, 5′-CGATACCAAAGTTGTCATGGA-3′.

### 2.3. Morphometric Analyses

The radial alveolar count (RAC) determines alveolar septation and is a test of alveologenesis. Through images at 100× magnification, a perpendicular line was made from a respiratory bronchiole to the nearest pleural edge or fibrovascular septum. Airspaces or saccules through this line were counted [22]. Scion Image software (Scion Corp., USA) was utilized to measure alveolar septal wall thickness [23].

### 2.4. Cell Culture and Treatment

Lung epithelial A549 cell line was commercially provided by ATCC (#CCL-185; USA) and was cultured in F-12 K Medium (#30-2004; ATCC) supplemented with 10% FBS. Human ATII cells and HEK-293 T cells were purchased from Procell (#CP-H209 and #CL-0005; Wuhan, China) and cultured in human ATII cell complete culture medium and DMEM, respectively. Cells were maintained in a 37°C incubator in the atmosphere of 95% and 5% CO_2_. A549 and ATII cells were exposed to different concentrations of O_2_ (21%, 40%, 60%, and 85%) in a standard modular chamber (#ENV-307A; Med Associates Inc., USA) at 37°C to assess the effects of hyperoxia on LTBR and CREB1 expression. The normoxia condition contains 21% O_2._ Based on the results of the preliminary assays, A549 and ATII cells were exposed to 85% O_2_ for 48 h to mimic the *in vitro* model of BPD. Si-NC, si-LTBR, si-CREB1, empty pcDNA 3.1, pcDNA 3.1-LTBR, and pcDNA 3.1-CREB1 were commercially provided by GenePharma (Shanghai, China). These oligonucleotides or vectors were transfected into A549 and ATII cells using Lipofectamine 3000 (Thermo Fisher Scientific, USA) for 24 h at 37°C. The transfection sequences used were as follows: si-NC: 5′-AACCATCACTTACAAGAAACC-3′; si-CREB1: 5′-GCTCGATAAATCTAACAGTTA-3′; si-LTBR: 5′-CCATCCATACTTCCCTGACTT-3′; pcDNA3.1: 5′-CATTGACGTCAATGGGAGTTTGTTTTGGCACCAAAATCAACGGGACTTTCCAAAATGTCGTAACAACTCCGCCCCATTGACGCAAATGGGCGGTAGGCGTGTACGGTGGGAGGTCTATATAAGCAGAGCTCTCTGGCTAACTAGAGAACCCACTGCTTACTGGCTTATCGAAATTAATACGACTCACTATAGGGAGACCCAAGCTGGCTAGCGTTTAAACTTAAGCTTGGTACCGAGCTCGGATCCACTAGTCCAGTGTGGTGGAATTCTGCAGATATCCAGCACAGTGGCGGCCGCTCGAGTCTAGAGGGCCCGTTTAAACCCGCTGATCAGCCTCGACTGTGCCTTCTAGTTGCCAGCCATCTGTTGTTTGCCCCTCCCCCGTGCCTTCCTTGACCCTGGAAGGTGCCACTCCCACTGTCCTTTCCTAATAAAATGAGGAAATTGCAT-3′; pcDNA 3.1-CREB1: 5′- ATGACCATGGAATCTGGAGCCGAGAACCAGCAGAGTGGAGATGCAGCTGTAACAGAAGCTGAAAACCAACAAATGACAGTTCAAGCCCAGCCACAGATTGCCACATTAGCCCAGGTATCTATGCCAGCAGCTCATGCAACATCATCTGCTCCCACCGTAACTCTAGTACAGCTGCCCAATGGGCAGACAGTTCAAGTCCATGGAGTCATTCAGGCGGCCCAGCCATCAGTTATTCAGTCTCCACAAGTCCAAACAGTTCAGATTTCAACTATTGCAGAAAGTGAAGATTCACAGGAGTCAGTGGATAGTGTAACTGATTCCCAAAAGCGAAGGGAAATTCTTTCAAGGAGGCCTTCCTACAGGAAAATTTTGAATGACTTATCTTCTGATGCACCAGGAGTGCCAAGGATTGAAGAAGAGAAGTCTGAAGAGGAGACTTCAGCACCTGCCATCACCACTGTAACGGTGCCAACTCCAATTTACCAAACTAGCAGTGGACAGTATATTGCCATTACCCAGGGAGGAGCAATACAGCTGGCTAACAATGGTACCGATGGGGTACAGGGCCTGCAAACATTAACCATGACCAATGCAGCAGCCACTCAGCCGGGTACTACCATTCTACAGTATGCACAGACCACTGATGGACAGCAGATCTTAGTGCCCAGCAACCAAGTTGTTGTTCAAGCTGCCTCTGGAGACGTACAAACATACCAGATTCGCACAGCACCCACTAGCACTATTGCCCCTGGAGTTGTTATGGCATCCTCCCCAGCACTTCCTACACAGCCTGCTGAAGAAGCAGCACGAAAGAGAGAGGTCCGTCTAATGAAGAACAGGGAAGCAGCTCGAGAGTGTCGTAGAAAGAAGAAAGAATATGTGAAATGTTTAGAAAACAGAGTGGCAGTGCTTGAAAATCAAAACAAGACATTGATTGAGGAGCTAAAAGCACTTAAGGACCTTTACTGCCACAAATCAGAT-3′ and pcDNA 3.1-LTBR: 5′-ATGGAAGCGACAGGAATCTCATTAGCATCTCAATTAAAGGTGCCTCCATATGCGTCGGAGAACCAGACCTGCAGGGACCAGGAAAAGGAATACTATGAGCCCCAGCACCGCATCTGCTGCTCCCGCTGCCCGCCAGGCACCTATGTCTCAGCTAAATGTAGCCGCATCCGGGACACAGTTTGTGCCACATGTGCCGAGAATTCCTACAACGAGCACTGGAACTACCTGACCATCTGCCAGCTGTGCCGCCCCTGTGACCCAGTGATGGGCCTCGAGGAGATTGCCCCCTGCACAAGCAAACGGAAGACCCAGTGCCGCTGCCAGCCGGGAATGTTCTGTGCTGCCTGGGCCCTCGAGTGTACACACTGCGAGCTACTTTCTGACTGCCCGCCTGGCACTGAAGCCGAGCTCAAAGATGAAGTTGGGAAGGGTAACAACCACTGCGTCCCCTGCAAGGCCGGGCACTTCCAGAATACCTCCTCCCCCAGCGCCCGCTGCCAGCCCCACACCAGGTGTGAGAACCAAGGTCTGGTGGAGGCAGCTCCAGGCACTGCCCAGTCCGACACAACCTGCAAAAATCCATTAGAGCCACTGCCCCCAGAGATGTCAGGAACCATGCTGATGCTGGCCGTTCTGCTGCCACTGGCCTTCTTTCTGCTCCTTGCCACCGTCTTCTCCTGCATCTGGAAGAGCCACCCTTCTCTCTGCAGGAAACTGGGATCGCTGCTCAAGAGGCGTCCGCAGGGAGAGGGACCCAATCCTGTAGCTGGAAGCTGGGAGCCTCCGAAGGCCCATCCATACTTCCCTGACTTGGTACAGCCACTGCTACCCATTTCTGGAGATGTTTCCCCAGTATCCACTGGGCTCCCCGCAGCCCCAGTTTTGGAGGCAGGGGTGCCGCAACAGCAGAGTCCTCTGGACCTGACCAGGGAGCCGCAGTTGGAACCCGGGGAGCAGAGCCAGGTGGCCCACGGTACCAATGGCATTCATGTCACCGGCGGGTCTATGACTATCACTGGCAACATCTACATCTACAATGGACCAGTACTGGGGGGACCACCGGGTCCTGGAGACCTCCCAGCTACCCCCGAACCTCCATACCCCATTCCCGAAGAGGGGGACCCTGGCCCTCCCGGGCTCTCTACACCCCACCAGGAAGATGGCAAGGCTTGGCACCTAGCGGAGACAGAGCACTGTGGTGCCACACCCTCTAACAGGGGCCCAAGGAACCAATTTATCACCCATGACTGA-3′.

### 2.5. CCK-8 Assay

A CCK-8 kit (#CA1210, Solarbio, Beijing, China) was applied to detect A549 and ATII cell viability. In brief, transfected cells were plated in 96-well plate and precultured in an incubator at 37°C and 5% CO_2_. Next, cells were added with 10 *μ*L of silencing or overexpressing plasmids. Ten *μ*L of CCK-8 solution was added, and then cells were cultured in the incubator for 2 h. OD value at 450 nm was read using a SpectraMax iD5 microplate reader (Molecular Devices, USA).

### 2.6. Western Blotting

Total protein was extracted from lung tissues and A549 and ATII cells using RIPA lysis buffer (#R0020; Solarbio). Protein concentration was measured with a BCA protein assay kit (#GK10009; GLPBIO, USA). Total protein (20~30 *μ*g/lane) was separated by 11% SDS-PAGE at 110 V for 2 h and transferred to 0.22 *μ*m PVDF membranes (Millipore, USA). The membranes were incubated with LTBR antibody (1 : 500, Abcam, ab70063), CREB1 antibody (1 : 1000, Abcam, ab32515), IKK*α* (phospho T23) antibody (1 : 500, Abcam, ab38515), IKK*α* antibody (1 : 1000, Abcam, ab32041), p52 antibody (1 : 10000, Abcam, ab175192), RELB antibody (1 : 2000, Abcam, ab235922), or GAPDH antibody (1 : 2000, Abcam, ab8245) at 4°C overnight. After washing with PBS, membranes were incubated with the secondary antibody IgG (1 : 2000, Abcam, ab6721) for 2 h at room temperature. Proteins were detected by enhanced chemiluminescence (#P0018S, Beyotime, Shanghai, China) based on the manufacturer's instructions. Protein band grey intensity was quantified using the Quantity One software (Bio-Rad, CA, USA).

### 2.7. Flow Cytometry

A549 and ATII cells were harvested, washed with PBS, and fixed with 1% paraformaldehyde overnight at 4°C. Next, cells were washed again, resuspended in 100 *μ*L 1 × Binding Buffer, and stained with 5 *μ*L Annexin V and 10 *μ*L PI using a commercial kit (40302ES50, YEASEN) for 15 min at room temperature in dark. Finally, the cells were resuspended in 400 *μ*L 1 × Binding Buffer, mixed on ice, and analyzed by FACS using flow cytometry (BD Biosciences, USA) within one hour. Cells were gated into four groups: Annexin V^−^/PI^−^, Annexin V^+^/PI^+^, Annexin V^+^/PI^−^, and Annexin V^−^/PI^+^. In this study, cell apoptosis rate was defined as the percentage of Annexin V^+^/PI^+^ cells (in late apoptosis stage).

### 2.8. Chromatin Immunoprecipitation (ChIP) Assay

This assay was performed with a ChIP assay kit (Beyotime, Shanghai, China) following the manufacturer's instructions. Briefly, A549 and ATII cells were cross-linked with 1% formaldehyde and sonicated to shear DNA to lengths between 200~1000 base pairs. Cell lysates were incubated at 4°C with protein A/G beads coated with the anti-CREB1 antibody (2 *μ*g, Abcam) or anti-IgG (2 *μ*g, Abcam) for one night. After washing and elution, samples were treated with 5 M NaCl for heating, and then incubated with proteinase K for 1 h. The bound DNA fragments were purified via DNA Extraction Kit (GeneMark, Shanghai, China) and analyzed by real-time PCR.

### 2.9. Luciferase Reporter Assay

Wild type (WT) LTBR gene promoter at different sites and the mutated (wt) sites were subcloned into the pGL3 luciferase reporter vector (GeneCopoeia). Mutation was performed using a QuickMutation™ Site-Directed Mutagenesis Kit (#D0206; Beyotime). HEK-293 T tool cells at the concentration of 5 × 10^6^ cells/well were transfected with pcDNA 3.1-CREB1 and the abovementioned pGL3 vectors containing LTBR gene promoter at different sites. Cell transfection was conducted using Lipofectamine 3000 reagent. Luciferase activity was measured with the Dual-Luciferase® Reporter Assay System (Promega).

### 2.10. Data Analysis

Data are presented as mean ± SD. For expression and luciferase activity values, data are represented as fold changes to mean control. For cell viability values, data are represented as percentage (%) of mean control. GraphPad Prism 8 (GraphPad Software, San Diego, CA, USA) was used to perform statistical tests including unpaired two-tailed Student's *t*-test and one-way ANOVA with Dunnett's or Tukey's post hoc test. A *p* < 0.05 was deemed as statistically significant. For *in vitro* studies, three biological replicates × three technical replicates were applied.

## 3. Results

### 3.1. LTBR and CREB1 Are Upregulated in Lungs of Hyperoxia-Stimulated Mice and in Hyperoxia-Treated A549 and ATII Cells

Hyperoxia-stimulated mouse model of BPD had lower body weight than normal mice (Figure 1(a)). Radial alveolar count values were lower, while alveolar septal wall thickness values were higher in hyperoxia-stimulated mice than normal controls (Figures 1(b) and 1(c)). Above assay results confirmed the successful establishment of the mouse model of BPD. Next, it was found that LTBR and CREB1 expression at mRNA and protein levels exhibited the upregulation in lungs of hyperoxia-stimulated mouse model of BPD (Figures 1(d) and 1(f)). There was a positive expression correlation between LTBR and CREB1 in lungs of hyperoxia-stimulated mice according to Pearson correlation analysis results (Figure 1(g)). Hyperoxia for 24 h and 48 h increased the expression of LTBR and CREB1 mRNA in A549 cells (Figure 1(h)). Their expression levels were concentration-dependently increased by O_2_ in A549 cells (Figure 1(i)). ATII cells were also used in this study. LTBR and CREB1 were also upregulated by hyperoxia in ATII cells (Figures 1(j) and 1(k)).

### 3.2. LTBR Silence Rescues the Influences of Hyperoxia on Viability and Apoptosis in A549 Cells

Two siRNAs, si-LTBR#1 and si-LTBR#2, were used to silence LTBR. LTBR expression was successfully decreased by si-LTBR#1/2 in A549 cells (Figures 2(a)–2(c)). Hyperoxia induced a significant decrease in cell viability and an obvious increase in apoptosis of A549 cells. Silencing of LTBR rescued the influences of hyperoxia on viability and apoptosis of A549 cells (Figures 2(d) and 2(e)).

### 3.3. LTBR Silence Increases Viability and Decreases Apoptosis in Hyperoxia-Stimulated ATII Cells

Si-LTBR#1 and si-LTBR#2 reduced LTBR mRNA and protein expression in ATII cells (Figures 3(a)–3(c)). LTBR silence rescued the negative influence of hyperoxia on viability and its positive influence on apoptosis of ATII cells (Figures 3(d) and 3(e)).

### 3.4. CREB1 Transcriptionally Activates LTBR

Si-CREB1 repressed CREB1 and LTBR protein expression in A549 (Figure 4(a)) and ATII cells (Figures 4(b) and 4(c)) regardless of hyperoxia. A ChIP assay was performed in A549 and ATII cells, confirming the binding of CREB1 protein and LTBR promoter (Figure 4(d)). We constructed the pGL3-LTBR promoter luciferase reporter vectors containing different sites of LTBR promoter and cotransfected these vectors with pcDNA-CREB1 into HEK-293 T tool cells. The results demonstrated that CREB1 showed very weak binding with the position -350~50 of LTBR promoter, while there was a significant binding of CREB1 on position -1100~ -600 of LTBR promoter (Figure 4(e)). A schematic map showed the potential binding of CREB1 on LTBR promoter (site 1 position -970~ -963: GGACGCCA and site 2-595~ -584: GCGGATGGCGCC, both predicted from the JASPAR database [24]), which was provided in Figure 4(f). The luciferase activity was repressed when both site 1 and site 2 were wild, as well as when site 1 or site 2 was mutated in A549 and ATII cells. At the same time, the luciferase activity was not changed when both site 1 and site 2 were mutated in A549 and ATII cells (Figure 4(g)). CREB1 significantly increased luciferase activity of pGL3 LTBR promoter site 1 and site 2 vectors in A549 and ATII cells (Figure 4(h)).

### 3.5. Si-LTBR Inactivates the NF-*κ*B Pathway

A previous study has shown that NF-*κ*B pathway is activated through the association of LTBR with TRAF2 and 3 [25]. Key proteins p-IKK*α*, IKK*α*, p52, and RELB involved in the NF-*κ*B pathway were assessed in A549 and ATII cells under the conditions of normoxia and hyperoxia. Hyperoxia increased the ratio of p-IKK*α*/IKK*α* and promoted p52 and RELB protein expression. Such effects were rescued by si-LTBR cotreatment (Figures 5(a) and 5(b)), indicating that silencing of LTBR suppressed the NF-*κ*B pathway.

### 3.6. Rescue Assays Assessing the CREB1/LTBR Axis in the Viability, Apoptosis, and NF-*κ*B Pathway-Associated Proteins in Hyperoxia-Stimulated A549 and ATII Cells

Rescue assays were conducted in hyperoxia-stimulated A549 and ATII cells. Si-LTBR rescued the repressive effect of pcDNA-CREB1 on the viability of hyperoxia-stimulated A549 and ATII cells (Figure 6(a)). Figures 6(b)–6(d) indicated that si-LTBR rescued the promotive effects of pcDNA-CREB1 on the apoptosis of A549 and ATII cells.  Figure 6(e) indicated that si-LTBR partially reversed the promotive influences of pcDNA-CREB1 on the ratio of p-IKK*α*/IKK*α* and p52 and RELB protein expression levels. Similarly, rescue effects of pcDNA-LTBR on si-CREB1 were explored. pcDNA-LTBR partially rescued the promotive effect of si-CREB1 on cell viability and its suppressive influences on cell apoptosis and NF-*κ*B pathway-associated key proteins in hyperoxia-stimulated A549 and ATII cells (Figures 7(a)–7(e)).

## 4. Discussion

Despite studies on LTBR in lung development or lung cancer [9, 26, 27], its role in BPD remains unknown. We used a mouse model of BPD by exposure to 100% O_2_ on postnatal day 4 followed by recovering for 10 days [19] and found that LTBR expression was increased in lungs of BPD mouse model compared with normal control mice. ATII cells are pulmonary epithelial progenitor cells and exist in the corners of alveoli, taking up only 5% of alveolar surface area in healthy adults with many functions including synthesizing and secreting surfactants, transporting intrapulmonary fluid and ion, supporting immune modulation, and regenerating alveolar epithelium after injury [28]. Injury of ATII cell is considered the key mechanism in BPD-related pulmonary epithelial injury [29, 30]. LTBR expression was also increased by hyperoxia-stimulated A549 and ATII cells in this study. Apoptosis of ATII is observed in hyperoxia-stimulated BPD model [19]. Our work supports that hyperoxia decreases cell viability and promotes apoptosis in A549 and ATII cells. However, hyperoxia-induced influences on A549 and ATII cells can be rescued by silencing of LTBR, indicating the protective role of suppressing LTBR in BPD.

CREB1 is a common transcriptional factor activated in lung injury, for example, activated CREB promotes expression of Lin28 in a mouse model of acute lung injury [31]. Endothelial cell-specific deletion of CREB1 induces lung vascular injury [32]. Hyperoxia induces DNA-hypermethylation of CREB1 promoter in lungs of newborn mice [33]. Proportion of ATII cells is significantly reduced in lungs of Creb1^−/−^ mice [34]. In our study, CREB1 protein expression levels were increased by hyperoxia in A549 and ATII cells. CREB1 transcriptionally activated LTBR in lung epithelial cells by binding to GGACGCCA and GCGGATGGCGCC in LTBR promoter. Consistent with our finding, previous studies also have revealed that CREB1 acts as a transcriptional factor to regulate gene expression, such as lncRNA CCAT1 [35] and GPX4 [36]. Moreover, CREB1 silence had the potential to increase A549 and ATII cell viability and decrease cell apoptosis, while such influence was partially restored by LTBR.

Multiple studies demonstrated that hyperoxia induced lung injury by activating the NF-*κ*B pathway in neonatal mice [37–39]. LTBR can induce the canonical and noncanonical NF-*κ*B signaling [11, 40]. We revealed the activation of NF-*κ*B pathway by hyperoxia in A549 and ATII cells and confirmed that LTBR silence suppressed the NF-*κ*B pathway. Knockdown of CREB1 can increase expression of phospho-NF-*κ*B p65 and NF-*κ*B p65 in human monocytes [41]. Some studies hold the opposite view that CREB1 activates the NF-*κ*B pathway [35, 42], which is consistent with our study. Our findings exhibited that CREB1 positively regulated the NF-*κ*B pathway by upregulation of LTBR. In addition, it has been reported that hyperoxia can induce lung injury via lung inflammation, leading to BPD [43]. NF-*κ*B is a common transcription factor associated with inflammation, leading to stimulation of inflammatory response and cell apoptosis [44]. Therefore, we speculated that CREB1 and LTBR might promote the NF-*κ*B pathway to affect inflammation in lung epithelial cells, and this conjecture will be explored in the further study.

Limitations of this study are addressed as follows: (1) expression data of LTBR in clinical lung tissues of BPD are lacked; (2) there is a close association of LTBR and WNT/*β*-catenin signaling [9], while this pathway was not included in this study.

In conclusion, this work innovatively demonstrated the upregulation of LTBR and CREB1 in BPD. LTBR and CREB1 are positive regulators of cell apoptosis and negative regulators of cell viability of A549 and ATII cells under hyperoxia. CREB1 induced LTBR expression at the transcriptional level to regulate NF-*κ*B pathway and further modulated lung epithelial cell viability and apoptosis. This study may aid in understating the pathogenesis and treatment of BPD.

## Figures and Tables

**Figure 1:** LTBR and CREB1 are upregulated in lungs of hyperoxia-stimulated mice and in hyperoxia-treated A549 and ATII cells. (a) Body weight of mice (in normoxia group and hyperoxia group) at postnatal day 14. (b) Radial alveolar count of mice. (c) Median alveolar septal wall thickness of mice. (d) Relative LTBR and CREB1 expression in lungs of hyperoxia-stimulated mouse model of BPD. PCR analysis was used. (e, f) LTBR and CREB1 proteins in lungs of BPD mice. Western blotting was used and relative grey density of LTBR was calculated using the ImageJ software. (g) Pearson correlation analysis was used to reveal expression correlation of LTBR and CREB1 in lung tissues of hyperoxia-stimulated mice. (h) Relative LTBR and CREB1 expression in A549 cells after exposure to 60% O_2_ for 24 h and 48 h. PCR analysis was conducted. (i) Relative LTBR and CREB1 expression in A549 cells after exposure to 21%, 40%, 60%, and 85% O_2_ for 48 h. PCR analysis was used. (j) Relative LTBR and CREB1 expression in ATII cells after exposure to 60% O_2_ for 24 h and 48 h. PCR analysis was performed. (k) Relative LTBR and CREB1 expression in ATII cells after exposure to 21%, 40%, 60%, and 85% O_2_ for 48 h. PCR analysis was used. ^∗^*p* < 0.05, ^∗∗^*p* < 0.01, ^∗∗∗^*p* < 0.001.

**Figure 2:** LTBR silence rescues the influences of hyperoxia on viability and apoptosis in A549 cells. (a–c) After transfection of si-LTBR#1 and #2 into A549 cells for 24 h, PCR and western blotting were used to examine the knockdown efficiency. (d) A CCK-8 kit was used to reveal A549 cell viability by various treatments. (e) An Annexin V-PI kit was used to reveal A549 cell apoptosis by various treatments. ^∗∗^*p* < 0.01, ^∗∗∗^*p* < 0.001.

**Figure 3:** LTBR silence increases viability and decreases apoptosis in hyperoxia-stimulated ATII cells. (a–c) PCR and western blotting were used to assess the knockdown efficiency of LTBR following 24 h transfection of si-LTBR#1/2 into human ATII cells. (d, e) A CCK-8 kit and an Annexin V-PI kit were used to detect ATII cell viability and apoptosis, respectively. ^∗∗∗^*p* < 0.001.

**Figure 4:** CREB1 transcriptionally activates LTBR. (a–c) Protein bands of CREB1 and LTBR in A549 and ATII cells under the condition of normoxia or hyperoxia and their corresponding quantitative graphs. (d) A ChIP assay was conducted in A549 and ATII cells. Relative enrichment of LTBR promoter in anti-CREB1 was assessed by PCR analysis. (e) A luciferase reporter assay was conducted in HEK-293 T tool cell line. Luciferase reporter vectors containing LTBR promoter fragments at sites of -100~50, -350~50, -600~50, -850~50, and -1100~50 were used. The empty luciferase reporter vector served as a control. (f) A schematic map to show the potential binding of CREB1 on LTBR gene promoter. Two DNA motifs of CREB1 were exhibited above CREB1. (g) A luciferase reporter assay was conducted in A549 and ATII cells. Luciferase reporter vectors containing wile type LTBR promoter sequences (-1100~50), LTBR promoter mutated A sequences (-1100~50, with GACGC mutated into CGACA in -969~ -965), LTBR promoter mutated B sequences (-1100~50, with GGATGG mutated into CATCCC in -593~ -588), and LTBR promoter mutated A + B sequences were used. (h) A luciferase reporter assay was conducted in A549 and ATII cells. Luciferase reporter vectors containing site 1 and site 2 and their flanking sequences were used. ^∗∗^*p* < 0.01, ^∗∗∗^*p* < 0.001.

**Figure 5:** Si-LTBR inactivates the NF-*κ*B pathway. (a, b) Protein levels of p-IKK*α*, IKK*α*, p52, and RELB in A549 and ATII cells were detected by western blotting. The ratio of p-IKK*α*/IKK*α* and relative grey density of p52 and RELB were shown in the graph bars following the protein bands. ^∗∗^*p* < 0.01, ^∗∗∗^*p* < 0.001.

**Figure 6:** Si-LTBR rescues the effects of pcDNA-CREB1 in the viability, apoptosis, and NF-*κ*B pathway-associated proteins in hyperoxia-stimulated ATII cells. (a) Cell viability of hyperoxia-treated A549 and ATII cells after transfection of pcDNA-NC, pcDNA-CREB1, and cotransfection of pcDNA-CREB1 + si-LTBR. (b, c) Flow cytometry results in A549 and ATII cells after indicated transfections. (d) Quantification analysis of the flow cytometry results in b and c to show cell apoptosis rate. (e) The ratio of p-IKK*α*/IKK*α* and relative grey density of p52 and RELB in hyperoxia-stimulated A549 and ATII cells were measured by western blotting. ^∗∗^*p* < 0.01, ^∗∗∗^*p* < 0.001.

**Figure 7:** Rescue effects of LTBR on si-CREB1 in the viability, apoptosis, and NF-*κ*B pathway in hyperoxia-stimulated ATII cells. (a) Cell viability of hyperoxia-treated A549 and ATII cells after transfection of si-NC, si-CREB1, and cotransfection of si-CREB1 + pcDNA-LTBR. (b, c) Flow cytometry results in A549 and ATII cells after indicated transfections. (d) Quantification analysis of the flow cytometry results in b and c to show cell apoptosis rate. (e) The ratio of p-IKK*α*/IKK*α* and relative grey density of p52 and RELB in hyperoxia-stimulated A549 and ATII cells were measured by western blotting. ^∗∗∗^*p* < 0.001.

## Data Availability

Data generated in this study are available from the corresponding author under reasonable requests.
